The article "Premarital Sexual Behavior among male college students of Kathmandu, Nepal" was retracted in 2023. Reason: lack of ethics approval or compliance.

# Premarital Sexual Behavior among male college students of Kathmandu, Nepal

**DOI:** 10.1186/1471-2458-9-241

**Published:** 2009-07-15

**Authors:** Ramesh Adhikari, Jyotsna Tamang

**Affiliations:** 1 Geography and Population Department, Mahendra Ratna Campus, Tribhuvan University, Kathmandu, Nepal; 2 Center for Research on Environment Health and Population Activities (CREHPA), Kathmandu, Nepal

## Abstract

**Background:**

In Nepal, as in other Asian countries, the issue of sexuality still remains a taboo. Despite this fact, an increasing number of sexual activities is being reported by Nepalese students. This trend warrants serious and timely attention. Due to the sensitivity of the topic of premarital sexuality, youth receive inadequate education, guidance and services on reproductive health. The main objectives of this paper are to explore the sexual behavior especially focusing on prevalence of premarital sex among college men and to investigate the factors surrounding premarital sexual behavior.

**Methods:**

A cross-sectional survey of college students was conducted in April-May 2006. A self-administered questionnaire was completed by 573 male students. Association between premarital sex and the explanatory variables was assessed in bivariate analysis using Chi-square tests. The associations were further explored using multivariate logistic analysis.

**Results:**

Despite the religious and cultural restrictions, about two-fifths of survey respondents (39%) reported that they have had premarital sex. The study has also shown that substantial proportions of students indulge in sexual activities as well as risky sexual behavior. Sex with commercial sex workers, multiple sex partners, and inconsistence use of condom with non-regular partner was common among the students. Less than two in five male students (57%) had used condom at the first sexual intercourse.

The prevalence of premarital sex varied on different settings. Older students aged 20 and above were more likely to have premarital sex compared with younger students aged 15–19. Men who had liberal attitude towards male virginity at marriage were almost two times more likely to have engaged in premarital sex compared to their counterparts who have conservative attitude towards male virginity at marriage. Moreover, those students who believe in Hindu religion were more than two times (OR = 2.5) more likely to have premarital sex compared with those who follow other religions. Furthermore, those men who have close unmarried friends who have experienced premarital sexual intercourse were eight times (OR = 8.4) more likely to be sexually active compared to those who did not have such sexually active friends.

**Conclusion:**

Prevalence of premarital sexual intercourse and risky sexual behavior are not uncommon in Nepal. Young people are exposed to health hazards due to their sexual behavior; hence sex education should be provided. School or college based sexuality education could benefit even out-of-school youths, because their partners often are students.

## Background

Nepal presents an important setting for addressing the sexual and reproductive health needs of young people as one-third of the country's population is aged 10–24 [1]. Data from the Central Bureau of Statistics also indicates that the percentage of never married people aged 10 and above is increasing over time (male 28% in 1961 to 39% in 2001; female 15% in 1961 to 30% in 2001) in Nepal [2].

In Nepal, as in other Asian countries, strong norms persist that prohibit premarital sexual contact between young men and women and the topic of sexuality largely remains a taboo. Due to decreased age at menarche and increasing tradition of later age at marriage, the customary attitude has been changing. Declining influence of family, increasing urbanization, migration and the exposure to mass media have collectively contributed to major changes in social and sexual behavior among adolescents [3]. Due to social restrictions, disclosure of premarital sexual activities is rare; however, few studies that have been conducted in Nepal indicate a growing trend towards premarital sexual activities among adolescents [4-6].

A study conducted by Tamang et al. in 1999 among Nepali men in the border towns of Nepal showed that a significant proportion of sexually experienced young unmarried (18–24 years) male who are residents of the border towns (54%) and non-residents (40%) had engaged in sex with a non-regular partner in the last 12 months preceding the survey. Higher proportion of the married non-resident young men (46%) compared with unmarried non-resident men (18%) were involved in casual sex and a large majority of the non-resident young men (67%) cited a commercial sex worker (CSW) as their last casual sex partner. Although regular use of condoms during sex with non-regular partners was generally low, only a small proportion of them considered themselves to be at risk of contracting sexually transmitted infections (STIs) and HIV/AIDS [5].

Another study of the young factory workers in Kathmandu revealed that 20% of unmarried boys and 12% of unmarried girls aged 14–19 years were sexually experienced (penetrative sex). Interestingly, the mean age for first sexual debut was the same for both the boys and the girls (15 years) [4]. Similarly a survey conducted among teenagers in seven districts of Nepal showed risky sexual behaviour especially among young boys. About 22% of the boys interviewed had premarital sexual experience and only two thirds of them used condom. The number of boys who had sex with multiple partners was also high [6].

Although nation wide and extensive research on young people's needs and behaviors in Nepal is rare, existing data indicate that young people do not have adequate access to appropriate information and services about sexual and reproductive health issues [4-6]. Even though young people are taught subjects on health and population at school levels which includes basic information on fertility, mortality, human organ, menstruation, sexually transmitted infections including HIV/AIDS, they are poorly informed about sexual and reproductive health mainly due to lack of comprehensive education about sexual and reproductive health [7]. The design and delivery of appropriate national level services for adolescents has been constrained by long-held traditional beliefs and ideologies. As a result of inadequate or ineffective services and information, young people often experience negative reproductive health consequences, including unplanned pregnancies and HIV/AIDS [3].

Many literatures suggest that the individual, family and peer variables have considerable influence on the sexual behavior of the youth. However, it is one of the least researched topics in Nepal. To fill the gap, it is thus imperative to study the factors surrounding premarital sex in the context of Nepal in order to inform policy makers and planners and to develop appropriate and timely intervention programs to prevent high risk sexual behavior such as premarital sex.

This article is based on a study conducted in 2006 in Kathmandu. Although the study was conducted among both male and female college students, the article focuses on data collected from male college students. The study sought to explore the sexual behavior especially focusing on prevalence of premarital sex among college men and to investigate the factors surrounding premarital sexual behavior. This study is the first of its kind conducted among college students. The findings of the study address the gap in knowledge by providing descriptive information on premarital sex that could help program managers of I/NGOs and the Government of Nepal to design appropriate and timely education-based interventions in institutions of secondary and higher education.

## Methods

The data used in this paper comes from a cross-sectional survey on attitude and behavior towards premarital sex among college students of Kathmandu Nepal carried out in 2006. Data for this paper was from 573 male students studying in 12 colleges affiliated to Tribhuvan University (TU) in Kathmandu, the capital of Nepal. The scientific committee which includes ethical review board of University Grant Commission (UGC) Nepal has approved the proposal and provided funding for this study.

Two-staged random sampling technique was applied in order to sample the college students. The first stage of sampling included random selection of 12 colleges affiliated to Tribhuvan University (TU) in Kathmandu. In order to select these 12 colleges, a list of all the private and public colleges affiliated to Tribhuvan University and those located in Kathmandu valley (includes three districts, namely Bhaktapur, Lalitpur and Kathmandu) was obtained from the office of the Vice Chancellor in Kathmandu. This list included colleges that provide intermediate (commonly known as Grade 11 & 12), undergraduate and graduate degrees. In the second stage, two classes were selected randomly from each sampled college. These classes were not differentiated by subject. The number of students in each class ranged from 40 to 60 students. Since all the colleges were co-educational, all male and female students present on the day of the interview in the sampled classes were requested to participate in the study. Female and male students were interviewed separately in different classrooms.

Due to the sensitive nature of the study, a self-administrated structured questionnaire (Additional file 1) was used to obtain information from the students. The questionnaires were first developed in English and then translated into Nepali language. The questionnaires were pre-tested among college students in a non-selected college and later refined as required. While most of the questions were close-ended, a few open-ended questions were also included.

The survey assessed four items that pertained to premarital sex: 1) Experience of sexual intercourse, 2) Age at first sexual debut, 3) First partner and 4) Use of condom during first sexual intercourse. Unmarried respondents were asked 'Have you ever had sexual intercourse?' and married respondents were asked 'Have you ever had sexual intercourse before you got married?'. These two questions were from two separate questionnaire items. In addition to this, the respondents were also asked about their age at first sexual debut, first partner and use of condom during first sexual intercourse.

All completed survey questionnaires were entered into a database after manual coding and validation. Data entry and validity checks were performed for all the questionnaires by using computer software dBase IV. The cleaned and validated data was transferred into SPSS for further processing and analysis.

Verbal informed consent was obtained from the participants before they were enrolled in the study. Consent form was written in the local language stating the study's objectives, nature of participant's involvement, risk and benefits, and confidentiality of the data. Students were requested to read the consent form carefully. They were given clear options on voluntary participation. It was also made clear that they could refuse to answer any questions and terminate the interview when they desired. None of the approached students refused to participate in the study. Confidentiality of information was ensured by removing personal identifiers from the completed questionnaires. The names of sampled colleges were not made public and thus not possible for anyone outside the research team to trace reported incidents of sexual behavior to respondents. Respondents were protected from any possible adverse repercussions of participating in the study.

Both bivariate and multivariate techniques were applied to identify the factors associated with the likelihood of having premarital sexual intercourse. Chi-square test was used to test an association between the variables. The variables were also examined in the multivariate analysis (Binary logistic regression) in order to identify the significant predictors after controlling for other variables. During the process of analysis, multi-collinearity among the variables was assessed and the least important variables were removed from the logistic model.

## Results

A large majority of the respondents (85%) were young (15–24 years). A large majority of the men (88%) were unmarried and 91 percent of sample students were from outside of Kathmandu valley. Students covered in this study were from 67 districts out of 75 districts of the country which means many (59%) lived either with friends or alone in Kathmandu (Table 1). More than half of the men were currently pursuing their undergraduate degree. Awareness of HIV/AIDS was universal among the male college students and knowledge of at least one mode of transmission of HIV/AIDS was also universal. A large majority of the students (91%) had taken up a subject in school or college related to reproductive health. Almost all students in the study reported that sex education is necessary for youth before getting married (table not shown).

**Table 1:** Selected background characteristics of the respondents

**Characteristics**	**%**
**Age group**	

15–19	35.8
20–24	49.2
25–29	12.7
30 and above	2.3
Median age	21.0

**Marital status**	

Unmarried	88.3
Currently married	11.7

**Districts**	

Kathmandu valley (3 districts)	9.2
Outside Kathmandu valley (64 districts)	90.8

**Level of education**	

Intermediate	27.7
Undergraduate	53.9
Graduate degree	18.3

**Type of accommodation**	

With family	41.0
Alone	19.0
With friends	40.0

**Total**	**100.0**
**N**	**573**

### Sexual Activities

The study shows a continuum of sexual behavior ranging from kissing, fondling to sexual intercourse. For example, more than half of the male (57%) had experienced kissing, while three-fifths of them (60%) reported that they placed their hand on a girl's breast. Similarly, more than a third (35%) reported that they placed their hand on a girl's sex organ. Dating in Nepali context seems to be less common compared to other non-penetrative sexual activities. Slightly less than half of the respondents (46%) reported that they experienced dating.

Overall, nearly half the men, both married and unmarried men (47%) had experienced sex while more than one third of the study respondents (39%) had premarital sex. Underreporting of such sexual activities is highly possible due to the sensitive nature of the study. Another proxy to measure experience of premarital sex is to ask if the respondent has close unmarried friend who has experienced premarital sex. As expected, more than half the respondents have a close friend who has had premarital sex (Table 2).

**Table 2:** Nature of sexual activities performed

	**%**
Experience of kissing a girl	57.4
Experience of dating	44.5
Experience of placing hand on a girl's breast	60.2
Experience of placing hand on a girl's sex organ	34.9
Experience of sexual intercourse	46.9
Experience of premarital sex	39.1
Having close unmarried friend with experience of premarital sex	53.0

**N**	**573**

Prevalence of premarital sex varied, depending on different settings. Slightly higher proportion of men in the age group of 20 years and above had premarital sex compared to younger men (below 20 yrs). Students who have higher education level reported higher percentage of premarital sexual experience. For example, around one third of men who were studying in intermediate level (35%) and more than two-fifths of students pursuing graduate degree (43%) had premarital sexual experience. Regarding marital status, higher proportion of unmarried men (40%) had premarital sex compared with currently married (33%) respondents. Similarly, level of premarital sexual activities is higher among those students whose permanent residence was outside Kathmandu valley (40%) compared with those who reside in Kathmandu permanently (32%).

Regarding living arrangement, the proportion of those students who lived alone had more premarital sex experience compared to others. For example, more than two-fifths of those men who lived alone (43%) had premarital sex while the percentage is less than two-fifths for those who live with family (37%).

Similarly, a significantly higher percentage of premarital sex was observed among students who have liberal attitude towards premarital sex compared to those who have conservative attitude towards the same. For example nearly half (46%) of the men who have liberal attitude towards female virginity (disagreed on the following statement: 'women should be virgin at marriage') had engaged in premarital sex. Similar response was found for the attitude towards male virginity (Table 3).

**Table 3:** Premarital sexual experience by selected background characteristics

	Premarital sex		Total	
	Yes	No	%	Number
**Age group**				
15–19	34.6	65.4	100.0	205
20 and above	41.6	58.4	100.0	368
**Level of education**				
Intermediate	35.2	64.8	100.0	159
Undergraduate	39.8	60.2	100.0	309
Graduate degree	42.9	57.1	100.0	105
**Marital status**				
Married	32.8	67.2	100.0	67
Unmarried	39.9	60.1	100.0	506
**District**				
Outside Kathmandu valley	39.8	60.2	100.0	520
Kathmandu valley	32.1	67.9	100.0	53
**Living arrangement**				
With family	36.6	63.4	100.0	232
Alone	43.4	56.6	100.0	106
With friends	39.6	60.4	100.0	235
Attitude towards female virginity***				
Conservative	33.4	66.6	100.0	305
Liberal	45.5	54.5	100.0	268
Attitude towards male virginity***				
Conservative	30.0	70.0	100.0	290
Liberal	48.4	51.6	100.0	283
**Family structure**				
Joint family	39.6	60.4	100.0	139
Nuclear family	38.9	61.1	100.0	434
Religion*				
Non-Hindu	20.0	80.0	100.0	35
Hindu	40.3	59.7	100.0	538
Has a friend who has experienced premarital sex***				
No	14.9	85.1	100.0	268
Yes	60.3	39.7	100.0	305

**Total**	**39.1**	**60.9**	**100.0**	**573**

Note: *** = p < .001, ** = p < .01, * = p < .05

Prevalence of premarital sex varied according to respondent's religion. For example, higher proportions of Hindu men (40%) were likely to have premarital sex compared to non-Hindu men (20%). It is also found that behavior of peers has positive effect on the prevalence of premarital sex. For instance, prevalence of premarital sex is far higher among those who have close unmarried friends with sexual experience (60% vs. 15%).

#### Age at First Sexual Intercourse

If unprotected, the first sexual event has clear adverse outcomes on health such as unplanned pregnancy for the women and STIs. Thus the first sexual intercourse remains an event of immense social and personal significance. In the current study, the age at first sexual intercourse of male students ranged from 10 to 25 years. About two-thirds of the respondents who had experienced premarital sex had sex before the age of 19. Seven percent reported that they had sexual intercourse before the age of 15 (Table 4).

**Table 4:** Age at first sexual intercourse

	**%**
Below 15 yrs.	6.7
15–16	25.0
17–18	32.0
19 or more	36.3

**Total (age range 10–25 years)**	**100.0**
**N**	**224**

#### First Sex Partner and Condom Use

Information regarding first sexual partner was solicited from students who had premarital sex. Over half the male students (55%) had their first sexual intercourse with their girlfriend while a third (32%) reported that their first sexual partner was their friend. It is notable that one out of ten male students (5%) had their first sexual intercourse with a commercial sex worker.

Condom use at the time of first sexual intercourse was very low. Less than three out of five students (57%) reported that they used condom during their first sexual intercourse.

### Sexual Risk Behaviour

#### Number of Sex Partners

Over half of the male students (55%) reported that they had more than one sex partner and about one in three sexually active men (31%) had three or more sex partners. The number of sexual partners for these college students ranged from 1 to 15 (Table 5).

**Table 5:** Number of sex partners

**How many sex partners did you have (total)?**	**%**
One	45.1
Two	23.7
Three and more	31.3
**Average number of sex partners**	**2.4**
**SD**	**2.1**
**Ranges**	**1–15**

**Total**	**100.0**
**N**	**224**

#### Sexual experiences with Commercial Sex Worker and Condom Use

Sexually active unmarried respondents were further asked about their sexual experiences with a commercial sex worker (CSW) and their condom use with them. The results show that more than a quarter of them (23%) had sexual intercourse with a CSW while only less than a half of the male students (49%) who had sexual intercourse with CSWs had used condom during every act of sexual intercourse (Table 6).

**Table 6:** Sex with CSW and condom use

	**%**
**Have you ever had sex with CSW?**	
Yes	22.8
No	77.2

**Total**	**100.0**
**N**	**224**

**How often did you use condom with CSW?**	
Every act of sexual intercourse	49.0
Sometimes	45.1
Never	5.9

**Total**	**100.0**
**N**	**51**

### Multivariate analysis

Logistic regression analysis was used to measure the strength of the association between various individual, family, peer's characteristics and the probabilities of being sexually active before marriage among these male students. Three models were used in the analysis. In the first model, individual factors were incorporated. In the second model, family characteristics were added and in the third model peer characteristics were included. After assessing multicollinearity in the variables, it was found that 'attitude towards male virginity at marriage' and 'attitude towards female virginity at marriage' were highly correlated (r = 0.8). So the variable 'attitude towards female virginity' was not entered in the logistic model.

The analysis found that men who have a liberal attitude (boys shouldn't be a virgin at marriage) towards male virginity at marriage were about two times more likely to have premarital sexual experience compared to those who have conservative attitude towards male virginity at marriage.

The variable which was significant in the first model retained significance even after inclusion of family characteristics in the second model. The reduction of odd ratio of the variable after inclusion of family characteristics indicated that the family characteristics were also important predictors for being sexually active among unmarried men. Model 2 further explained that those students who believe in Hindu religion were about three times (OR = 2.6) more likely to have premarital sex compared to those who believe in the Muslim religion (Table 7).

**Table 7:** Estimated odds ratio (OR) for having premarital sex among college-going men by selected predictors

	**Model I**	**Model II**	**Model III**
**Individual characteristics**			
**Age group**			
15–19	1.0	1.0	1.0
20 and above	1.34	1.39	1.69*
**Level of education**			
Intermediate	1.0	1.0	1.0
Undergraduate	0.93	0.89	0.52*
Graduate degree	0.88	0.79	0.48*
**Marital status**			
Married	1.0	1.0	1.0
Unmarried	1.30	1.29	1.73
**District**			
Outside Kathmandu valley	1.0	1.0	1.0
Kathmandu valley	0.82	0.84	0.97
**Living arrangement**			
With family	1.0	1.0	1.0
Alone	1.32	1.39	1.28
With friends	1.05	1.07	1.07
**Attitude towards male virginity**			
Conservative (ref)	1.0	1.0	1.0
Liberal	2.16***	2.15***	1.91**
**Family characteristics**			
**Family structure**			
Joint family		1.0	1.0
Nuclear family		0.91	0.81
**Religion**			
Non-Hindu (ref)		1.0	1.0
Hindu		2.63*	2.99*
**Peer characteristics**			
**Has close unmarried friend who has experienced premarital sex**			
No (ref)			1.0
Yes			9.2***
Intercept	0.28	0.124	0.033
-2 log likelihood	741.7	736.1	611.1
Cox & Snell R square	0.043	0.052	0.238

Note: *** = p < .001, ** = p < .01, * = p < .05

Model three presents the final results after adding peer characteristics. Even after inclusion of peer characteristics in the third model, the individual variable and one family-level variable were still statistically significant. Furthermore, the variables 'age', 'level of education', 'having close unmarried friends who have had premarital sex' had statistical significant effect on experience of premarital sex after controlling for other variables. Older students aged 20 and above were about two times (OR = 1.7) more likely to have premarital sex compared with younger students aged 15–19. Unexpectedly, those students who have studied undergraduate and graduate degree level of education were less likely to have premarital sex compared with those who have intermediate education only. Those men who had close unmarried friends who had experienced premarital sex were almost eight times more likely to be sexually active compared with those who did not have such friends (Table 7).

## Discussion and conclusion

This study is first of its kind in Nepal and attempted to investigate the influencing factors surrounding premarital sexual behavior among college men. Although premarital sex is socially unacceptable in Nepal, the study has shown that the proportion of students having sexual intercourse before marriage is considerably high. Due to the sensitive nature of the issue, this proportion may still be underreported. However another variable in the study shows that more than half of the college students have friends who have had premarital sexual experience. This variable is an indication of the high prevalence of premarital sex among college male students.

The study also showed that risky sexual behavior is common among college men. Condom use at the time of first sexual intercourse was very low among these men. More than a quarter of the male students (23%) had had sexual intercourse with a commercial sex worker. Although awareness about HIV/AIDS and mode of transmission of HIV/AIDS were universal among the male students, it is discouraging to note that only less than half the students (49%) who had sexual intercourse with CSWs had used condom at every act of sexual intercourse, which indicates these sexually active men are more at risk

The increase in premarital sex among men who are attending school/college may be due to the fact that they have greater independence (not living with family) from their families and increasing access to young women for sex. The prevalence of premarital sex varied with different settings. The bivariate analysis showed that some of the individual characteristics, family variables and peer characteristics had significant association with experience of premarital sex. Individual characteristics such as attitude towards male and female virginity, family characteristics such as religion and peer characteristic such as peer sexual behavior have significant association with having premarital sex among college-going men. The multivariate analysis corroborated some of the findings of the bivariate analysis. In the multivariate analysis, age, attitude towards male virginity, religion and peer sexual behaviour were found to have statistical significant association with experience of having premarital sex after controlling for other variables.

The association between age cohort and premarital sex is substantial. The present study found a positive association between age cohort and premarital sex, but it cannot be concluded that the likelihood of premarital sex is declining among the younger cohort; the association is undoubtedly an artifact of the truncated exposure among the younger cohort. Research has shown that young people who identify with a fundamentalist Protestant group have less permissive attitudes toward premarital sex and these young people are likely to be less sexually active [8]. The present study also supported this finding as students who have liberal attitudes toward premarital sex were more likely to engage in premarital sex. However, some of the students who had conservative attitude had also engaged in premarital sex. One of possible reason for this finding could be peer pressure.

Peer role is important in changing personality, attitude and behavior of persons. There is further evidence that in all societies, peer behavior is a model for individual behavior, and this is certainly true in matters of sexuality among adolescents and youths [9]. Even in the present study, the sexual behavior of the peer was positively associated with premarital sex.

Sometimes peer pressure upon a person can lead him or her to engage in sex through associated behaviors such as drinking alcohol and seeking CSWs. A study showed that two thirds of the men perceived that after drinking with friends, refusal to visit a brothel upon their friends' request has caused misunderstanding with them [10]. Similarly another study among school aged adolescents in Kenya (1993) showed that males who socialized with sexually experienced peer were nearly seven times more likely to have sex than those whose peers were not sexually experienced [11]. Sensitive issue such as sexuality is difficult to discuss among family members but it is easier to discuss among peers. Therefore, the impact of peer group plays a significant role in influencing views, attitudes and sexual behavior of individuals. Although this paper presents a worthy picture regarding premarital sexual behavior, it cannot be generalized to all college students in Kathmandu valley as the sample was taken only from those colleges that are under the umbrella of Tribhuvan University. Furthermore, since the study was conducted among college students, it also excludes an important group such as out-of-school individuals.

In short, we would like to summarize that many findings from our study are in line with findings from previous studies on premarital sexual behavior. This paper not only provides empirical evidence on the importance of individual characteristics, familial role and peer factors on premarital sexual behavior of male college students in Nepal, but also draws attention to the prevalence of premarital sexual behavior among young, college-going youths. This paper seeks to fill the gap in knowledge by providing descriptive findings on premarital sex among college male students and to garner interest from policy-makers to develop appropriate reproductive health programs to combat negative impact of such behavior. Our findings suggest that it is necessary to reinforce reproductive and sexual health education among college students and provide them with convenient and optional services that are easily accessible. There is a need to provide comprehensive education on sexual and reproductive health (SRH) issues such as safer sex and HIV/AIDS in order to make responsible and healthy decisions to protect them from situations and behaviors that would place them at risk of HIV transmission. It is further recommended that a qualitative research should be conducted in order to design appropriate intervention that address the problems and needs of the youths by involving the young people themselves.

## Competing interests

The authors declare that they have no competing interests.

## Authors' contributions

RA, Lecturer of Mahendra Ratna Campus, Tahachal, Kathmandu conceived and designed the study. He carried out the data collection, conducted data analysis and interpretation of the data. JT was involved in the data analysis and interpretation of the datav.

## Pre-publication history

The pre-publication history for this paper can be accessed here:



## Supplementary Material

Additional file 1 **Questionnaire on the study entitled "Survey on Attitude and Behavior towards premarital sex among college students of Kathmandu Valley"**. The questionnaire includes various aspects of information regarding premarital sex. Click here for file
